# Advances in CRISPR/Cas9

**DOI:** 10.1155/2022/9978571

**Published:** 2022-09-23

**Authors:** Youmin Zhu

**Affiliations:** School of Economics and Management, Qiannan Normal College for Nationalities, 558000, China

## Abstract

CRISPR/Cas9 technology has become the most examined gene editing technology in recent years due to its simple design, yet low cost, high efficiency, and simple operation, which can also achieve simultaneous editing of multiple loci. It can also be carried out without using plasmids, saving lots of troubles caused by plasmids. CRISPR/Cas9 has shown great potential in the study of genes or genomic functions in microorganisms, plants, animals, and human beings. In this review, we will examine the history, structure, and basic mechanisms of the CRISPR/Cas9 system, describe its great value in precision medicine and sgRNA library screening, and dig its great potential in a new field: DNA information storage.

## 1. Introduction

Gene editing technology refers to the operation method of modification of designated DNA target sequence in the genome to achieve DNA fragment knockout, insertion, or other sequence changes. In the early stage of gene editing, homologous recombination was used to achieve sequence exchange between two DNA strands with homology. This technology is, however, inefficient and error-prone. Later, Meganuclease, ZFNs, and TALEN were developed through artificial modification of nuclease and used for gene editing [1–3]. The modified nuclease is a chimera consisting of a specific DNA binding domain and a non-specific DNA cleavage domain [4, 5]. These technologies solved the key problem of gene editing: to create double-strand breaks (DSBs) at specific sites of genome. However, the binding domain sequences need to be redesigned each time when identifying different sites. Additionally, the design of the constructs is complex and the experimental process is tedious [6]. Compared to the previous gene editing technologies, CRISPR/Cas9 technology has been proved to be more efficient in construction, which was consequently quickly applied into production [7]. The sustainable improvement of the CRISPR/Cas9 system has realized great application value in gene function research, gene therapy, and genetic improvement, allowing the research in Life Sciences to reach new heights.

## 2. The Discovery of the CRISPR/Cas9 System

The repetitive tandem arrays were initially discovered in *Escherichia coli* (*E. Coli*) in 1987 [8]. There are a series of highly conserved DNA repeats in bacterial and archaeal genomes, which are separated by interspaced sequences [8]. It was later found that about 40% of bacterial genomes and 90% of archaeal genomes contain these unique sequences [6, 9]. In 2002, this unique family of repetitive tandem arrays was officially named clustered regularly interspaced short palindromic repeat (CRISPR) [9]. Subsequently, the CRISPR-associated protein (Cas), which is nuclease or helicase being functionally related to CRISPR, was discovered [10, 11]. The CRISPR sequences are homologous with phage sequences and the homology can reach up to 100% [9, 12]. This indicates that the CRISPR sequences may be derived from phage. In 2005, three research groups found that CRISPR may be related to the immunity of microorganisms [11–13], which led scientists to pay closer attention to CRISPR. The researchers speculated that CRISPR might be involved in the defense mechanism of bacteria [11–13]. They hypothesized that the CRISPR could use antisense RNA to memorize and recognize the exogenous nucleic acids invading cells. This defense mechanism is similar to the RNAi mechanism of eukaryotic self-immune function [14]. The self-immune function mediated by CRISPR/Cas system was soon proved in an experiment using Lysozyme to infect *Streptococcus thermophiles* [15]. CRISPR/Cas is believed to be the “acquired immune system” evolved by bacteria or archaea in the process of resisting foreign DNA from plasmids or phages [7, 16].

## 3. The Basic Structure of the CRISPR/Cas9 System

CRISPR/Cas system can be divided into three types: type I, type II, and type III. Type I and type III are relatively complex. However, the type II CRISPR/Cas system of *Streptococcus pyogenes SF370* is very simple, which only involves Cas proteins. Cas9, in particular, is a ~160KD protein with six domains (Rec I, Rec II, Bridge Helix, RuvC, HNH, and Protospace Adjacent Motif interacting (PI)) which can independently target and cleave DNA [6, 7]. Due to its simplicity, type II CRISPR/Cas9 system has become a powerful tool for gene editing after being improved [17–19]. The type II CRISPR/Cas locus consists of a trans-activating CRISPR RNA (tracrRNA) region at the 5′ end, a series of *Cas* genes (*Cas9*, *Cas1*, *Cas2*, and *Csn2*) encoding proteins essential for immune response, and a CRISPR region at the 3′ end which consists of a large number of spacers and direct repeats [6] (Figure 1). tracrRNA (encoded by the tracrRNA region) and crRNA (CRISPR RNA, encoded by the CRISPR region) form crRNA : tracrRNA complex to achieve specific DNA sequence recognition.

The nuclease encoded by *Cas* gene is guided by crRNA to achieve site-specific DNA cleavage. Two important components of *Streptococcus pyogenes* Cas9 (spCas9) protein are recognition (REC) lobe and nuclease (NUC) lobe. REC lobe consists of a long alpha helix and two REC domains, REC1 and REC2, which are the functional domains of spCas9 when interacting with repeat: anti*-*repeat duplex. NUC lobe consists of PI, RuvC nuclease, and HNH nuclease domains [21]. HNH domain is located at the amino terminal of spCas9 protein, which is responsible for cleaving the DNA sequence complementary to crRNA. The cleavage site is located at the third nucleotide upstream of the Protospace Adjacent Motif (PAM) [17, 22, 23]. RuvC domain interacts with sgRNA through a surface with positive charges produced by the interaction of RuvC domain and PI domain. sgRNA is a short artificial RNA that can replace crRNA to guide spCas9 protein to cleave target DNAs at specific site [24]. REC lobe first combines with sgRNA to search for PAM sequence on the target DNA. Then, sgRNA can be paired with the target DNA to guide the RuvC and HNH domains in NUC lobe to cleave the two strands of the target DNA. HNH domain cleaves the DNA strand recognized by sgRNA, while RuvC domain cleaves the complementary strand. A groove with positive charges, which is formed between REC lobe and NUC lobe, is the region where sgRNA guides spCas9 to cleave the target DNA [25, 26]. The PAM is an important component for targeting [7], whose main function is to help Cas9 accurately distinguish its own DNA and foreign DNA with identical sequence. This indirectly protects its own DNA from attack by nuclease, so as to achieve targeted cleavage of foreign DNA [6, 27]. Cas9 protein is inactive in its own presence; however, when Cas9 is combined with sgRNA, the conformation of Cas9 protein will change dramatically, enabling Cas9 to be activated to cleave the target DNA [25, 26] (Figure 2).

## 4. The Mechanism of the CRISPR/Cas9 System

The process of bacteria resisting the invasion of foreign nucleic acids mainly includes three stages: adaptation, expression, and interference [6, 29]. When a virus invades a bacterium for the first time, the bacteria will digest the virus DNA into spacer sequences with proper sizes by recognizing its specific PAM sequences and integrate them into its CRISPR spacer region, enabling the bacteria to memorize the invading virus [30]. When invaded by the same kind of virus again, the bacteria are able to recognize it and transcribe the spacer sequences into pre-crRNA. The pre-crRNA will be paired with tracrRNA and be processed into mature crRNA with the help of CnsI and RNaseIII [31]. crRNA recognizes and binds the foreign DNA through complementary sequences; thus, this crRNA is also called guide RNA (gRNA) [32]. Cas nuclease cannot cleave the foreign DNA by itself; however, when combined with a mature tracrRNA and crRNA to form the ribonucleoprotein complex, Cas protein can be guided by crRNA to cleave the invading DNA by recognizing its PAM site so as to destroy the foreign DNA and achieve self-defense [33, 34].

The specific target sequence recognition ability of crRNA, the DNA cleavage activity of Cas nuclease, and the DNA repair mechanisms of cells endow the CRISPR/Cas system with the function of gene editing. When DSBs occur, cells will activate their own repair mechanisms to repair DNA damage and avoid cell death. There are two repair mechanisms: non-homologous end joining (NHEJ) and homology-directed repair (HDR) [35, 36]. If homologous sequences are available, the cells normally activate HDR mechanism to repair DSBs by homologous recombination, which is to integrate homologous fragments into DNA. Utilizing this repair mechanism, we can artificially design a repair template (donor) DNA fragment with homologous arms and co-transform it with gene editing vector, allowing integration of donor DNA into cell genomic DNA to achieve gene knock-in [37]. When homologous DNA is not available, the cells normally initiate NHEJ mechanism, which links the broken DNA directly. This repair mode is prone to base pair insertions or deletions (indels) that may generate gene frameshift mutations resulting in gene knockout [38, 39] (Figure 3).

In gene editing, Cas9 and gRNA can be constructed into one vector or two different vectors equipped with corresponding promoter, terminator, replicon, and selection marker. The artificially designed gRNA is a chimeric RNA containing a combination of all the essential crRNA and tracrRNA components [40]. The front portion of the gRNA is called sgRNA which is responsible for recognizing the target site. The following part functions as a scaffold for binding to Cas9 protein [7]. sgRNA is required to be modified each time when identifying different targets. The preferable length of sgRNA is 20 nt, making it easy to construct CRISPR/Cas9 vector. As a potential target can be found in every 8 bp DNA sequences on average, there are many potential targets suitable for CRISPR/Cas9 [34]. These factors have enabled the CRISPR/Cas9 system to be the most popular tool for gene editing. When CRISPR/Cas9 vectors are transformed into target cells, they will express Cas9 and gRNA which can perform gene editing [6]. In 2013, CRISPR/Cas9 was used for gene editing in eukaryotic cells for the first time. Scientists successfully edited *Th* gene of mice as well as *EMX1*, *PVALB*, *PPP1R12C*, *CLTA*, and *CCR5* of human beings using CRISPR/Cas9 [41–43]. Thereout, the gene editing function of CRISPR/Cas9 was confirmed. The simplicity of the CRISPR/Cas9 system has consequently attracted a large number of scientists to exploit it in-depth, making it one of the biggest scientific breakthroughs in the last decade.

## 5. The Application of the CRISPR/Cas9 System

### 5.1. CRISPR/Cas9 Gene Editing in Microorganisms, Plants, and Animals

Gene knockout, gene insertion, and other DNA sequence modifications mediated by CRISPR/Cas9 technology may generate changes in gene expressions or phenotypes of living organisms, making CRISPR/Cas9 technology a vital method for gene function research, character modification, and new life substance production. Gene modification using CRISPR/Cas9 technology has been applied in many microorganisms, plants, and animals and plays a significant role in strain improvement as well as crop and livestock breeding.

There are many kinds of microorganisms which are widely distributed and play important roles in agriculture, industry, and medicine. In 2013, CRISPR/Cas9 gene editing was used in bacteria for the first time [32]. Due to the lack of endogenous NHEJ pathway, most bacteria can only repair DSBs through HDR [44, 45]. Therefore, in addition to Cas9 protein and gRNA, a template for HDR is needed in bacteria. The repair template/donor can be either a single-strand DNA (ssDNA) or double-strand DNA (dsDNA) [46]. A ssDNA donor, however, has a higher efficiency than dsDNA for DSBs repair [47]. In order to improve the efficiency of recombination in bacteria, *λ*-Red recombination system or RecET system should be introduced into host cells [20, 48]. Otherwise, the exogenous NHEJ system needs to be introduced into the bacteria to fill in for the lack of NHEJ repair [49–51]. Cas9 and gRNA can be expressed by a single plasmid, double plasmid, or multiple plasmid systems [52]. The single plasmid system contains all the necessary elements including gRNA, Cas effector protein (CEP), and donor, achieving target site cleavage and repair in a single round transformation [53]. In addition, an appropriate CEP should be selected for gene editing in bacteria, because CEP may be toxic to host cells [20, 54]. Recently, researchers used CRISPR/Cas9 technology to edit *Streptococcus mutans* for gene function study [55], which can assist in speeding up the understanding of novel species. CRISPR/Cas9 technology has also been successfully used to edit the genome of *Saccharomyces cerevisiae* (*S. cerevisiae*) [27]. Furthermore, researchers have fused 16 chromosomes of yeast into one or two chromosomes using CRISPR/Cas9 technology. The modified yeast showed only a slight growth defect [56, 57], indicating future possibilities of using CRISPR technology to break the boundaries of nature and even artificially create new lives that do not exist in nature.

In plants, gene editing has been successfully carried out in Arabidopsis (*A. thaliana*), tobacco (*Nicotiana tabacum L.*), rice (*O. sativa*), and wheat (*Triticum aestivum L.*) to improve crop yield, quality, or stress resistance [58, 59]. Researchers knocked out the *TaMLO* gene of hexaploid wheat using CRISPR/Cas9 technology and obtained a new wheat line resistant to Powdery Mildew [60]. A pure herbicide-resistant rice line was obtained using CRISPR/Cas9 to replace two amino acid residues at the same time in *ALS* gene [61]. Soyk et al. used CRISPR/Cas9 technology to edit *SP5G*, a gene that can inhibit flowering of tomato, which accelerated flowering and ripening, significantly increasing its yield [62]. Zhang et al. used CRISPR/Cas9 system to knock out *Clpsk1* gene, the precursor of plant sulfonylkinase (PSK), which weakened plant immune response and enhanced the resistance of watermelon to *Fusarium oxysporum f.* sp. *niveum* (FON) [63]. Gao *et al.* obtained a waxy corn line by editing its 12 waxy alleles using CRISPR/Cas9. The waxy corn was also found to be superior to the hybrids in agronomic trait and yield [64]. Jia and Wang likewise used CRISPR/Cas9 to produce homozygous anti-ulcer orange in T0 generation [65]. The application of CRISPR/Cas9 technology in plants has thus enabled plant gene function research and crop genetic improvement to develop rapidly.

Gene editing has been successfully carried out in animals from the lower *Caenorhabditis elegans* [66] to the higher primate *Cynomolgus monkeys* [67]. In 2013, three laboratories successfully knocked out a single gene, double genes, and multigenes of mouse cells, respectively, using CRISPR/Cas9 technology [34, 39, 58]. Scientists have also used D10A–Cas9–nickase technology to modify chicken primordial germ cells to produce a myostatin*–*knockout (MSTN*–*KO) chicken, which significantly increased the skeletal muscle of its chest and legs [68]. It is really a great piece of news for KFC and all who like eating chicken. Researchers are also trying to redesign and manufacture livestock through CRISPR technology in order to increase animal husbandry production to meet the growth of human demand for food and reduce the adverse impact on the global environment [37].

### 5.2. Precision Medicine

A prominent reason as to why scientists are very much interested in gene editing is due to its potential use in precision medicine. Gene editing carries the hope of curing many genetic defects and other severe illnesses that could not be treated by conventional therapy. At present, CRISPR/Cas gene editing has been successfully utilized in mammalian models, which is of great significance to precisely and accurately observe phenotypes and pathogenesis, better understand pathophysiology, promote gene therapy to a greater extent, and present new opportunities for the development of new treatment methods. Wu et al. cured cataract mice by injecting Cas9 and sgRNA into the fertilized eggs of mice with cataract pathogenic gene (*CRYGC*) mutation [69]. Yin *et al.* successfully cured genetic tyrosinemia caused by *Fah* gene mutation using CRISPR/Cas technology [70]. These researches verified the feasibility of precision medicine mediated by CRISPR/Cas. In 2014, the CRISPR system was delivered into the liver of adult mice via tail vein injection for the first time to knock out two primary tumor suppressor genes, *p53* and *PTEN*, generating a mouse liver tumor model [71]. In 2016, Kang et al. used CRISPR/Cas9 technology to knock out the *RUNX3* and *IL2RG* genes of pigs and constructed a human gastric cancer model [72]. Shortly after, the CRISPR system was successfully used in brain, lung, and liver disease models [73]. Chang *et al.* found a safe knockout site in monkey embryonic kidney epithelial cells (Marc*–*145 cells) using CRISPR/Cas9 technology, which has potential use in increasing vaccine production in the future [74].

The knockout of HIV receptor *CCR5* in HIV-infected human blood T cells or CD4 hematopoietic stem cells can effectively reduce the virus level and improve the survival rate of CD4 cells [75–77]. Ye et al. knocked out the 32 bp sequences of *CCR5* of multifunctional stem cells using CRISPR/Cas9 technology to effectively block the invasion of HIV [78], proving the effectiveness of using CRISPR/Cas9 to edit cell receptor for the treatment of HIV and other viral diseases. Ebina et al. and Hu *et al.* used CRISPR/Cas9 technology to edit the cells with integrated *HIV–1* genes and successfully restricted the activation and replication of the virus by generating mutations at the *HIV–1* fragments [79, 80], opening up a new way for HIV treatment. Eliminating HIV will, however, turn AIDS into a chronic disease as its genes can integrate into the genome of the infected person. The result is that the infected person will have to be on medication for his entire life instead of receiving a viable cure. A favorable option is to combine CRISPR technology with existing antiviral drug therapy, that is to use antiretroviral drugs to inhibit the replication of the virus while using CRISPR/Cas9 technology to remove the HIV DNA fragments integrated into the genome [81, 82]. Conceivably, the use of CRISPR/Cas technology alone may not be an absolute cure for AIDS without the assistance of antiretroviral drugs. However, when CRISPR/Cas9 technology combines with CRISPR/Cas13a technology which can target RNA virus, it may eliminate the *HIV–1* gene integrated into the human genome and kill the virus simultaneously.

Gene editing has made a great breakthrough in antitumor immunotherapy. Chimeric antigen receptor T cell immunotherapy (CAR*–*T cell immunotherapy) is one of the most sought-after immunotherapies for oncotherapy. Chifman et al. used CRISPR/Cas9 technology to obtain modified T cells which recognizes specific receptors on tumor cell surface, preventing tumor cells from immune escape and enhancing their defense ability against tumor cells [83]. Wu *et al.* used CRISPR/Cas9 technology to eliminate endogenous T cell receptor genes and human leukocyte antigen I (*HLA I*) of biological immune T cells while importing the CAR sequence, producing universal CAR*–*T cells that were applied to patients and dismissed the possibility of host immune rejection [84–86]. Inhibition of gene expression involved in the negative regulation of immunity could also achieve antitumor effects. Knocking out the *PD–1* gene of T cells using CRISPR/Cas9 technology can prevent the impact of immune regulators on the activation and proliferation of T cells, improving T cell activities against tumor cells [87, 88]. Researchers have also used CRISPR/Cas9 technology to remove *CD33* from hematopoietic stem cells in AML patients, leaving CD33+ cancer cells as the only target of CD33 CAR*–*T cells [89]. Additionally, CRISPR/Cas9 was used to knock out the *BCL–6* gene in Diffuse Large B-cell Lymphoma (DLBCL), which resulted in stagnation of cell cycle (G1) in tumor cells, bringing hope for curing this disease [90]. Zhen and Kennedy et al. edited the human papillomavirus genome to explore the potential of CRISPR/Cas9 technology in preventing cervical cancer caused by papillomavirus [91, 92]. Zhang *et al.* have recently applied CRISPR/Cas9 technology to gynecological cancer treatment [63] which presents a probable breakthrough in gynecological cancer treatment. These studies prove that CRISPR/Cas9 technology can be used to develop safe and effective tumor-targeted therapies.

CRISPR/Cas9 could effectively edit haploid mutations of human embryonic stem cells, providing a new way in the study of human genes, especially those in recessive alleles [93]. Scientists used CRISPR/Cas9 technology to remove herpesvirus and hepatitis B virus genomes and explored the potential of CRISPR/Cas9 technology in the treatment of chronic infectious diseases [94–96]. Liao et al. activated the expression of endogenous *PDX1* with CRISPR/dCas9 in diabetic mice to induce secretion of insulin which can effectively treat diabetes [97]. Long *et al.* used CRISPR/Cas9 technology to correct the muscle and cardiac abnormalities associated with DMD [98]. Researchers also used CRISPR/Cas9 technology for the first time to treat a patient blinded by Leber's congenital amaurosis 10 (LCA10), a rare genetic defect. This clinical trial is a milestone in gene therapy as the disease was not curable by any other means [99]. Besides treating diseases, CRISPR/Cas9 technology has the potential to change the aging process to prolong human life [100]. For these reasons, the application of the CRISPR/Cas system is worth being examined more extensively for the future benefit of humanity. The CRISPR/Cas system may be utilized to remedy all incurable diseases and maintain physical health conditions.

### 5.3. sgRNA Library

sgRNA library screening technology is a powerful tool for systematic genomic analysis. It is an important research method to study gene, RNA, and protein functions; quickly screen for drug targets and quickly breed new varieties of animals, plants, and microorganisms. The main existing sgRNA libraries include CRISPR knock-out, knock-in, activation, and inhibition libraries, which can achieve high-throughput screening of the whole genome. Tens of thousands of sgRNA covering the whole or part of the genome are designed and synthesized on a chip. The sgRNAs are then recombined into appropriate vectors to construct plasmids which are monitored by high-throughput sequencing. After being packaged by lentivirus, plasmids are transformed into host cells to introduce various gene mutations. Finally, candidate genes are identified by observing the phenotypic changes of host cells. Presently, scientists have successfully constructed many human and mouse genomic libraries which are still under continuous improvement [101]. Yilmaz et al. generated 180,000 different mutations using sgRNA library to screen and analyze all genes in the human genome, drawing a blueprint of the human genome and revealing the roles of the genes in disease occurrence [102], which is of great significance for the treatment of many human diseases. Most of the sgRNA libraries were screened by *in vitro* culture or cell transplantation models. Recently, however, researchers have achieved *in vivo* screening of cells and targets, enabling the rapid generation of patient-specific avatars to guide precision medicine [103]. The construction of sgRNA libraries in multi-species promotes the development of biological research and produces much economic value.

### 5.4. Gene Editing without Plasmids Remained

Plasmids are usually transformed into target cells for CRISPR/Cas9 gene editing. The plasmids which remain in the cells after transformation will, however, lead to adverse effects on subsequent experiments. Persistent expression of Cas9 will increase the risk of off-target [104]. Moreover, the selective marker of the plasmids prevents researches from employing subsequent plasmids with the same marker next time. If we can eliminate the plasmids after or in the process of gene editing, the above problems will be solved. A definite solution is to transform the Cas9 protein and the gRNA, both expressed *in vitro*, directly into target cells. Another solution is to transform the plasmids into target cells to achieve gene editing before transforming a transcribed gRNA targeting the plasmids into the cells to remove the plasmids. Due to the high cost of gRNA transcription *in vitro*, researchers have developed other methods, such as adding a temperature-sensitive replicator in the plasmids to eliminate the plasmids by changing the temperature after gene editing [52, 105, 106]. Besides that, a target DNA fragment can be placed into the plasmids for the sgRNA to guide the Cas9 protein to target and remove the plasmids while gene editing is being done.

### 5.5. Cas9 Modifications

Only when both HNH and RuvC domains of wild-type Cas9 protein function normally can they create DSBs in the genome. However, when one of the domains is inactive, Cas9 turns into Cas9 nickases (Cas9n), which can only cause single-strand breaks (incisions). Cas9n can be selected to carry out heterozygous editing, when editing some homozygous lethal genes. Another application of Cas9n is that it can be used as a base editor when combined with deaminase and DNA polymerase. By fusing Cas9n with deaminase, site-specific cytosine/thymine or adenine/guanine mutation will be introduced into the incision created by Cas9n during the repair process mediated by DNA polymerase [107–110]. When both HNH and RuvC domains are inactive, Cas9 turns into dead Cas9 (dCas9), which has the function of binding rather than cleaving DNA [111]. dCas9 can be used to activate or inhibit the transcription of genes via binding to transcription regulator*-*binding sites, which technique is called CRISPRa or CRISPRi [111–114]. This technique promotes functional gene screening and identification of genes for specific diseases [115]. Furthermore, dCas9 can be used for fluorescence imaging when combined with fluorescent proteins to observe the dynamic changes of the DNA or trace some interesting DNA sites.

### 5.6. Other Applications

In addition to the above, CRISPR/Cas9 technology plays vital roles in SNP detection and multiplexed CRISPR editing. The site-specific recognition and incision in CRISPR/Cas9 technology are employed to detect SNP as the sgRNA designed at the SNP site will only recognize a specific genotype, allowing different genotypes to be distinguished. The application of the CRISPR/Cas9 system in DNA detection has, as such, promoted basic biology and applied biology research [116]. Another advantage of CRISPR/Cas9 is in its use for multigene editing by linking several distinct gRNAs in one plasmid to target and edit different sites simultaneously [60]. When constructing tandem gRNAs, a promoter can be placed in front of each gRNA. Another good alternative is to connect gRNAs through tRNAs. As tRNA is very short, it will keep the plasmid from becoming too big, to avoid any effect in the transformation efficiency. On top of that, tRNA is comparable to an enhancer, which can promote the expression of the far-end gRNAs. Zhang et al. used gRNA*–*tRNA array to edit *S. cerevisiae* genome, knocking out 8 genes at the same time and achieving 87% efficiency [117]. Using double gRNAs to target two sites on the same chromosome which are far away from each other may lead to large segment deletion [118]. Recently, researchers eliminated the direct repeats (DRs) through Reversed Paired*–*gRNA Plasmid Cloning Strategy to resolve the problem of instability of double gRNAs in the same direction, realizing the rapid deletion of 100 kb chromosome segment in *E. coli* [119]. Multiple CRISPR technology has extensive application prospects in cellular recorders, genetic circuits, biosensors, combinatorial genetic perturbations, large-scale genome engineering, and the rewiring of metabolic pathways [120].

## 6. Off-Target Effect

CRISPR/Cas9 technology is not perfect. It has its deficiency, one of which is the off-target effect. Finding out the reasons for the off-target effect is the key to reduce the off-target rate. When sgRNA recognizes the target DNA by complementary base pairing, the matching of the sgRNA and the DNA shows tolerance to a certain degree. The sgRNA designed for the target may consequently recognize a wrong site which is highly homologous to the target DNA sequence, as there are many similar sequences in the large complex genome, resulting in an unexpected gene editing in the wrong site. The entire genome sequencing of mice cells showed that there were a high number of mutations after editing by CRISPR/Cas9 [121]. The off-target effect of CRISPR/Cas9 has been demonstrated in functional studies of plant genome [109, 122] and clinical applications [123–125], indicating the CRISPR/Cas9 system's off-target effect to be a widespread phenomenon. There are two main kinds of mismatches between sgRNA and the target DNA. One is that the sequence length of the sgRNA is the same as the off-target site, but with a few bases mismatched [126, 127]. The other is where a few bases of differences between the length of the sgRNA and the off-target site led to a partial base pairing and form a hairpin shape structure [128]. The length of the hairpin structure can reach to 5 bp [128]. Off-target effect may bring some experimental troubles or even wrong results or phenotypes, which seriously restricts the application of CRISPR/Cas9 technology.

## 7. Safety and Ethical Issues

The news of the birth of the world's first gene-edited babies, who are assumed to be resistant to AIDS, has caused a huge stir all over the world. It is a typical example of how humans would change the genetic code of a human body to meet human desires and needs. This may encourage parents to alter their children's genes according to their values, resulting in genetic inequality after birth. There are also safety issues in gene editing due to the lack of thorough research on the CRISPR/Cas9 system and the risk of off-target effects that could lead to unpredictable consequences in the future. Researchers have used gene editing technology to eliminate some genes that could cause immune rejection in T cells, to prevent the patients' immune system and anticancer drugs from attacking foreign T cells, expecting to improve patients' immune ability and cure leukemia [129]. However, it was later discovered that DSBs caused by CRISPR/Cas9 could kill human pluripotent stem cells [130, 131]. Recently, researchers have found that Cas9 can interact with KU86 subunit of DNA-dependent protein kinase (DNA*–*PK) complex to prevent the NHEJ pathway from repairing DSBs. The Cas9 variants, Xcas9 and dCas9, can also interact with KU86 to disrupt DSBs repair. In consideration of the decisive role of DNA*–*PK to maintain genomic stability and the effect of DSBs on cell proliferation and survival, there are pressing safety concerns in the clinical application of the CRISPR/Cas9 system [132]. With the rapid development of the CRISPR/Cas9 technology, the scope and extent of its application should be strictly monitored and evaluated to minimize the side effects.

## 8. Directions for Future Developments of the CRISPR/Cas9 System

### 8.1. Improvements in Editing Efficiency

One of the main future directions in the development of the CRISPR/Cas9 system is to improve its editing efficiency. In addition to the multi-CRISPR system, several more methods, such as the internal sequence optimization of the CRISPR/Cas9 system, delivery system improvement, and changing DNA repair strategy, are being implemented to improve the editing efficiency. The internal sequence optimization of the CRISPR/Cas9 system includes modification of sgRNA sequence, target sequence selection, PAM sequence redesign, Cas9 sequence modification, and promoter selection. The modification of the sgRNA sequence enhances its activity to recognize the target site and achieve gene editing with fewer designed sgRNAs. Choosing an appropriate target site facilitates the design of optimal gRNA for target recognition. PAM sequences also affect the efficiency of gene editing. Generally, the efficiency of NGG is higher than the NGA and NAG [133]. Zhang et al. compared 16 different PAM sequences and found that the cutting efficiency of Cas9 for NGG was 2 and 4 times higher than that of NGA and NAG, respectively [134]. As Cas9 supposedly required PAM for DNA incision, this limited the choice of targets to some extent. Recently, however, Walton et al. designed two Cas9 protein variants, SpG and SpRY, which could bind and cleave DNA without specific PAM, indicating there were potential targets throughout the genome [135]. Xing *et al.* discovered that optimizing Cas9 codon could improve the gene editing efficiency of maize [136]. Using different promoters to initiate the expression of Cas9 or gRNA can also affect the editing efficiency. *TaU3* promoter, for example, was found to be more efficient in initiating the gRNA transcription in maize [136]. Furthermore, the development of new biological delivery systems (such as particle bombardment delivery, electric pulse and electromagnetic radiation delivery, and nanotechnology delivery systems) has increased the editing efficiency through the improvement of the transformation efficiency [29, 137–139]. Recently, researchers developed a single “All*–*in*–*One” Helper*–*Dependent Adenovirus (HDAd), which could deliver donor DNA, Cas9, and sgRNA to achieve efficient gene targeting and HDR repair simultaneously [140]. Additionally, inhibiting the efficiency of NHEJ to increase HDR efficiency could also improve the efficiency of gene editing [141].

### 8.2. Reduction of Off-Target Effects

Many people doubt CRISPR/Cas9 technology due to its off-target effect, which presents severe issues in therapeutics as it generates loss-of-function mutations in proper functional genes or incorrect repairing of disease-inducing genes [142]. Reducing the off-target rate of CRISPR/Cas9 has thus been one of the main priorities. Cas9n, which can only cut a single DNA strand, has been observed to reduce the off-target effect. Two designed sgRNAs, one for the DNA sense strand and another for the antisense strand, can be used to target adjacent sites, enabling gene editing to occur only when the two sgRNA*–*Cas9n systems work simultaneously [43, 143–145]. This method is, however, limited by PAMs. Being inspired by Cas9n, Tsai et al. designed the Fok1*–*dCas9/gRNA complex, a combination of dCas9/gRNA and Fok1, and found that two concurrent Fok1*–*dCas9/gRNA complexes with adjacent target sites on the two strands of DNA generate DSBs [146]. Furthermore, using a new small nuclease Cpf1 instead of Cas9 could achieve higher accuracy and lower off-target effect [147]. The specificity of the CRISPR/Cas9 system mainly depends on the sgRNA. Many biotechnological companies are consequently developing sgRNA design software. With the support of bioinformatics and big data, biotechnological companies can automatically carry out whole genome comparison and select the sgRNAs with low off-target rate. There are various sgRNA online design software on the market at present, including CRISPR*–*FOCUS, CHOPCHOP, and CRISPR library designer (CLD) [101]. Xiao et al. invented the CasOT tool, which could identify potential off-target sites in the whole genome to help reduce the off-target rate [147]. The study found that the 10*–*12 nt of the 20 nt sgRNA carried out the primary function of target recognition, while the 8*–*10 nt sequences played a secondary role [18, 20, 35]. Therefore, the key to reducing the off-target rate is to ensure the specificity of the 10*–*12 nt [18]. The length and the sequence characteristics of the sgRNA may also affect the off-target rate. Researchers have developed a number of CRISPR/Cas9 variants, including sgRNAs ranging from 17 nt to 24 nt. Studies showed that shortening the 20 nt sgRNA to 17 nt [148] or adding two guanine nucleotides to the 5′ end of sgRNA could reduce the off-target rate [127, 149, 150]. Using an 18 nt sgRNA instead of a 20 nt sgRNA could effectively reduce the risk of off-target in mammalian cell editing [148]. The long-lasting high-intensity expression of Cas9 could significantly increase the off-target rate. However, a lower concentration of Cas9 could reduce the off-target rate by weakening the cutting capacity of the endonuclease [127]. The off-target effect is relatively low when the ratio of gRNA: Cas9 is between 2 : 1*–*3 : 1 [104]. Additionally, the GC content of the sgRNA was also found to correlate with the off-target effect, enabling researchers to select more effective sgRNAs by their GC content [134]. Moreover, using Cas9 mRNA or protein instead of plasmids could also effectively reduce the off*-*target rate [151, 152]. A mutant of Cas9, xCas9, is more precise than Cas9, can effectively reduce the off-target rate, and has been successfully used in gene therapy [153]. The cutting efficiency of Cas9 sometimes varies according to the characteristics of the PAM sequences [81]. Choosing the right PAM site can reduce the off-target effect. Cell types could also affect the off-target effect [154]. Selecting the most appropriate cell type may help improve the accuracy of gene editing and diminish the off-target effect.

### 8.3. Medicine Production

The CRISPR*–*Cas9 system has become a remarkably powerful technique for the treatment of human disease. One promising field is to use CRISPR*/*Cas9 technology to produce medicine. An example is to use the CRISPR/Cas9 system to genetically modify some antibodies thus producing new antibodies with higher affinity to antigens. Recently, the genomes of sheep and goats were modified using CRISPR/Cas9 to express the medicine in their mammary glands, making it a shortcut for medicine production [155].

### 8.4. DNA Information Storage

In recent years, a new scientific field involves the combination of CRISPR/Cas9 technology with synthetic biology to conduct DNA information storage. The exponential growth of digital information in this era has made traditional information storage methods redundant due to limitations in capacity and density, poor durability, and high maintenance cost. To develop a new storage media with higher density and better durability is one of the research frontiers in the field of digital information storage [156]. Compared with existing magnetic and optical storage media, DNA has the advantages of better durability, higher storage density, and environmental protection [157]. It is estimated that one cubic inch of DNA can store all the electronic data in the world [158]. DNA is highly stable and can be preserved for 1 million years at *–*18°C [159], allowing it to undoubtedly be the best choice for information storage in the future. After transforming digital information into DNA information, we can use CRISPR/Cas9 technology to insert the synthesized DNA into the genome to achieve high-density storage as well as information replication through the reproduction of the organism [160].

CRISPR/Cas9 technology has greatly promoted the development of many biological fields due to its high efficiency and simplicity. A high biological safety is achieved as it eliminates the position effect of the traditional transgenic technology. Researchers can modify a few base pairs rather than inserting a complete gene into the genome, which will ease public concern. The potential of CRISPR/Cas9 has, however, not been fully explored, as our understanding of the CRISPR/Cas9 system is still limited. Further improvement of the CRISPR/Cas9 system may bring more surprising discoveries and application value.

## Figures and Tables

**Figure 1:** CRISPR/Cas9-mediated bacterial adaptive immunity. A typical type II CRISPR/Cas locus consists of a set of *Cas* genes (colored ellipses), a series of repeats (yellow diamonds) and spacers (green rectangles). When phages infect a cell, the cell will capture and integrate the phages' DNA fragments into the CRISPR array. Spacers are then transcribed into crRNA precursor (pre-crRNA) (brown line) and paired with tracrRNA (blue line) to be cleaved into mature crRNA by RNase III. crRNA recognizes foreign DNA through complementary pairing and guides Cas9 to make site-specific DNA breaks on foreign DNA [20].

**Figure 2:** The overall structure of the Cas9 protein and the schematic diagram of the Cas9–sgRNA-target DNA complex in a type II CRISPR/Cas system. Cas9 protein comprises NUC and REC lobes. REC lobe contains a long alpha helix and two REC domains. NUC lobe consists of PI, RuvC, and HNH domains. RuvC and HNH domains have cleavage functions, which can recognize the PAM site and cut the target DNA under the guide of the crRNA: tracrRNA complex [25, 28].

**Figure 3:** CRISPR/Cas9-mediated NHEJ and HDR. When DSBs occur, cells will use the NHEJ or HDR mechanism for DNA repair. The NHEJ mechanism will directly link the broken DNA together and can be utilized for gene knockout. The HDR mechanism repairs the broken DNA by homologous recombination and can be utilized for gene knock-in [37].
